The article "Association of Frailty Status and Functional Disability among Community-Dwelling People Aged 80 and Older in Vietnam" was published in 2021. Journal: Biomed Res Int.

# Association of Frailty Status and Functional Disability among Community-Dwelling People Aged 80 and Older in Vietnam

**DOI:** 10.1155/2021/7109452

**Published:** 2021-07-19

**Authors:** Thu Thi Hoai Nguyen, Anh Trung Nguyen, Thanh-Huyen Thi Vu, Nga Thi Dau, Phong Quy Nguyen, Thanh Xuan Nguyen, Tam Ngoc Nguyen, Huong Thi Thu Nguyen, Thang Pham, Huyen Thi Thanh Vu

**Affiliations:** ^1^Hanoi Medical University, Hanoi 100000, Vietnam; ^2^National Geriatric Hospital, Hanoi 100000, Vietnam; ^3^Dinh Tien Hoang Institute of Medicine, Hanoi 100000, Vietnam; ^4^Feinberg School of Medicine, Northwestern University, 60611, USA

## Abstract

**Objectives:**

This study investigated associations between frailty and functional disability in elder suburban Vietnamese.

**Method:**

Cross-sectional analysis was carried out on 251 participants aged 80 and over in Soc Son district. We used the Instrumental Activities of Daily Living (IADL) scale including 8 items, and functional disability was defined as ≥3 IADL impairment. We defined frail as ≥3 out of 5 frailty components including weight loss > 5%, weak grip, exhaustion, low walking speed, and low physical activity.

**Results:**

Of 251 participants with a mean age of 84.6, 11.2% was classified as frail and 64.5% had ≥3 IADLs. Among the frailty components, low walking speed and low physical activity were significantly associated with increased odds of having ≥3 IADLs: ORs (95% CI) were 4.2 (2.3-7.9) and 3.7 (1.7-8.2).

**Conclusion:**

Frailty is associated with the higher likelihood of having functional disability. Further longitudinal studies are needed to examine the causal this relationship.

## 1. Introduction

Vietnam's population is ageing rapidly. The proportion of people aged 80 and older currently is over 2 million [1, 2]. While showing success in improving life expectancy, the ageing population raises many social issues, particularly the healthcare for older people. This issue should be given more concern in order to reduce the incidence of functional disability, multimorbidity, and mortality [3].

Frailty is defined as a common and important geriatric syndrome characterized by age-associated declines in physiologic reserve and function across multiorgan systems, leading to increased vulnerability to adverse health outcomes including falls, incident disability, hospitalization, and mortality [4, 5]. Previous studies have indicated that the prevalence of frailty in communities varies significantly (range 4.0-59.1%) [6, 7]. Indeed, social, intellectual, biological, and functional factors play an important role in the development of frailty [8]. A certain number of clinical conditions are associated with frailty and the onset of functional decline in older people [9–12]. Moreover, in people aged 80 and over, frailty is correlated with a higher risk of adverse health outcomes, including functional disability. Previous studies have suggested that functional disability can be measured by the changes in ability to perform Instrumental Activities of Daily Living (IADLs) [13]. This instrument is commonly used in communities and various epidemiological studies [14, 15].

The article "Association of Frailty Status and Functional Disability among Community-Dwelling People Aged 80 and Older in Vietnam" was published in 2021. Journal: Biomed Res Int.

The Vietnamese government has started to support a universal minimum pension for people aged 80 and older since 2011. Therefore, maintaining the functional ability of older people and screening early decline will reduce the financial burdens and improve the quality of life of an ageing population [16]. Understanding the characteristics, prevalence, and potential risks of frailty is essential for initiating adequate and cost-effective intervention programs in older adults. There is abundant research on frailty, but it is limited in Vietnam, especially on the association of frailty and functional disability in Vietnamese people aged 80 and above. Data on functional disability and frailty from Vietnam can provide useful insights for developing appropriate policies and programs for the elderly in communities. Therefore, this paper proposes to investigate the association between frailty and functional disability among older people.

## 2. Methods

### 2.1. Study Setting

This cross-sectional study was conducted in 2016 in Soc Son district, a suburban area located in northern Hanoi with a population of approximately 330,000 people. This is a noncommercial agriculture area with ease of access to medical services.

### 2.2. Sample Size and Sampling

A formula for a proportion with a specified relative precision was used to calculate the sample size. With the confidence interval of 95% and a relative precision of 0.05, the expected prevalence of frailty in the community was 12.3% [17]. The minimum sample size was 166. All people aged 80 years and over living in 5 communes in Soc Son district were invited to participate in the study. In total, 996 invitations were sent to older people aged ≥80 years old, 299 people came (30%), and 251 participants completed the questionnaire and assessment.

### 2.3. Data Collection

Data were collected through a personal household interview conducted by well-trained field workers and nursing students, who were trained during two days in both the class room and field setting. Data quality was controlled in the field by supervisors as well as by the investigators of this study.

### 2.4. Measurements

#### 2.4.1. Frailty Syndrome Assessment

The Fried frailty phenotype [9] including five criteria with some adaptations was used to define frailty in all participants, including unintentional weight loss > 5% per year, weak grip strength (measured with a dynamometer, and the highest value of both hands was used), exhaustion (“In this last month, do you feel that you have less energy to do the things you want?”), low walking speed (the cut point of 5 seconds after walking 4 m), and low physical activity (“How often do you practice any of the following activities (dancing, walking, farmer work, or gardening)?”). Participants who met at least three criteria were considered frail, whereas those with one or two criteria were prefrail and those with no characteristics were defined as robust [9].

The article "Association of Frailty Status and Functional Disability among Community-Dwelling People Aged 80 and Older in Vietnam" was published in 2021. Journal: Biomed Res Int.

#### 2.4.2. Functional Disability Definition

The Instrumental Activities of Daily Living (IADL) questionnaire [13] included 8 items (using telephone, shopping, food preparation, housekeeping, laundry, mode of transportation, responsibility for own medications, and ability to handle finances) and was used to evaluate the capabilities of performing daily activities with tools [18]. Each IADL item was scored as impaired (score = 0) or not (score = 1); hence, the summary score ranges from 0 to 8. Functional disability based on the summary score was dichotomized as ≥3 IADL disability (1 = Yes, 0 = No).

#### 2.4.3. Health-Related Data

Height (cm) and weight (kg) were measured and BMI was calculated [19]. BMI then was classified as underweight (BMI < 18.5 kg/m^2^), normal weight (BMI from 18.5 to 22.9 kg/m^2^), and overweight (BMI ≥ 23 kg/m^2^) [20]. Current drinking alcohol (Yes/No) and any chronic diseases such as hypertension, diabetes, COPD, Parkinson, and stroke were also included in the analysis.

*Other covariates* included age, sex, educational level (uncompleted high school < 12 years of schooling), high school graduated (12 years of schooling), studying college and higher (>12 years of schooling), marital status (married, single, widow, or divorced), occupation (farmer, retired), and living status (living with children, living alone, or living with caregivers).

### 2.5. Statistical Analysis

Both descriptive and analytical statistics were carried out using Stata software (version 14.0). Proportions or means (standard deviation, SD) were calculated for all participants and compared across frailty categories using *F* tests for continuous variables or chi-square tests for categorical variables. Multivariable logistic regression modelling was performed to examine the association between frailty and functional disability. A significance level of *p* < 0.05 was used. Models were adjusted for age, gender, education levels, marital status, occupation, BMI levels, and current status of drinking alcohol and chronic disease. The analyses were performed for the combined-component frailty and functional disability and then for single components (i.e., 5 frailty components and 8 IADL items).

The article "Association of Frailty Status and Functional Disability among Community-Dwelling People Aged 80 and Older in Vietnam" was published in 2021. Journal: Biomed Res Int.

### 2.6. Ethical Approval

The study protocol was approved by the institutional review board of the National Geriatric Hospital (Reference number: 35/QD-BVLKTW). Participants were asked to give their oral informed consent. The information was kept confidential and used only for research purposes.

## 3. Results

Table 1 summarizes sociodemographic characteristics, health behaviors, and health status, as well as the prevalence of functional disability of the study sample, overall and by frailty category. Among 251 participants, 28 (11.2%) participants were frail and 127 (50.6%) prefrail. The mean age of all respondents was 84.6 (4.2) years, and 68.5% were female. Age, sex, education, body mass index level, and smoking were significantly associated with the frailty status with *p* value < 0.05. With regard to the prevalence of functional disability, there were 64.5% of disability with ≥3 IADL items.

Figure 1 shows the prevalence of individual frailty components of the study sample. Low walking speed was most prevalent (41.4%) and weight loss was least prevalent (8.0%).

Figure 2 presented the prevalence of participants having disability ≥ 3 IADL items and by component. The item most frequently reported was telephone use (70.9%), and there were 64.5% of disability ≥ 3 IADL items.

Logistic regression analysis found a statistically significant association between frailty status and functional disability (assessed in combination (≥3 IADLs vs. otherwise) or singly (impaired vs. not impaired), i.e., for 8 items separately) (Table 2). With adjustments for age, sex, education, marital status, occupation, BMI levels, current drinker, and having any chronic disease, frailty was associated with having three or more disabilities in IADLs. Compared to those with a robust health condition (0 frailty component), the odds (95% CI) of having ≥3 IADL disability in frail and prefrail participants were 9.0 (2.5-34.3) and 2.9 (1.6-5.3), respectively. Similar results were observed for associations between frailty status and individual IADL items, except for the inability to use the telephone (Table 2).

Among frailty components, low walking speed and low physical activity were significantly associated with increased odds of having ≥3 IADL disability when compared to their counterparts (Table 3): adjusted ORs (95%) were 4.2 (2.3-7.9) and 3.7 (1.7-8.2), respectively. Although the results were not statistically significant, those with weight loss > 5%, weak grip strength, or exhaustion still had higher odds of having functional disability (higher by 14-43%) (Table 3).

The article "Association of Frailty Status and Functional Disability among Community-Dwelling People Aged 80 and Older in Vietnam" was published in 2021. Journal: Biomed Res Int.

## 4. Discussion

Among 251 participants aged 80 years and over in a suburban area of northern Hanoi, Vietnam, the prevalence of frailty was about 11%, and 64.5% had ≥3 IADL disability. Associations existed between frailty status and disability, with frailty being associated with having ≥3 IADL disability. Frailty was also associated with all individual disability items except for telephone-use impairment. These associations were independent of participants' sociodemographic characteristics, behaviors, and health conditions. Low walking speed and low physical activity were main components of frailty that were significantly associated with increased odds of having disability.

The prevalence of frail people in our study was higher than the prevalence of frailty in the Fried study (6.9%) [9] and Wu et al. study (7%) [21]. The participants in our study, however, were older than those in the Fried and Wu et al. studies. The prevalence of frail people in our current study was lower than the prevalence of a previous study (35.4%) conducted in inpatient participants in Vietnam using the same Fried criteria [22].

The prevalence of having ≥3 IADL disability items was 64.5% in our study, which was significantly higher than in the study of community-dwelling older women aged over 75 years by Nourhashémi et al. (9.5%) [13]. The most likely explanation for this difference is that the people in our study are aged 80 and over.

Our finding is consistent with those from previous studies that functional disability is a strongly associated with frailty [6]. Early screening and preventing adverse health outcomes from frailty are essential. Due to the lack of studies on this issue in Vietnam, this study was important to provide more information. Therefore, it is necessary to inform policy makers and healthcare workers about frailty among the older in community dwellings. Moreover, because low walking speed and low level of physical activity have a strong association with IADL disability, healthcare workers should focus on physical activity in frail people. Encouraging useful exercises and suitable activities for older people is necessary to minimize the risk for functional disability. Long-term plans and early screening for frailty and intervention should be considered to reduce the adverse outcomes of frailty. As the prevalence of frailty and functional impairment among community-dwelling people aged 80 and older in suburban Vietnam are relatively high, increasing the awareness of healthcare providers towards the importance of functional assessment of frail people is necessary.

The article "Association of Frailty Status and Functional Disability among Community-Dwelling People Aged 80 and Older in Vietnam" was published in 2021. Journal: Biomed Res Int.

### 4.1. Strength and Limitations

To our knowledge, our study is the first in Vietnam reporting the relation of frailty with disability in an older suburban population. This pilot study assesses the association between frailty and disability in IADLs among people aged 80 and older in community-dwelling areas of suburban Vietnam. This study will contribute to the literature on frailty and functional decline of Vietnam's older population. However, the study has several key limitations. First, this is a cross-sectional study; thus, causal inferences cannot be established. Second, being a pilot study, it is not representative of all people aged 80 and over in Vietnam. Finally, there should be differences in culture and lifestyles between suburban Vietnam and Western countries; hence, the adaptation of IADL measurements should be considered. For example, telephone use or shopping may not be common activities for suburban Vietnamese aged 80 and over. An adaptation regarding cultural and geographical differences of IADL measurements is needed in future research in Vietnam.

## 5. Conclusion

In summary, our findings contribute to the developing literature on the relationship between frailty and disability in older Vietnamese. Given that the proportion of frailty and functional disability in people aged 80 years and over in community-dwellings was relatively high, increasing awareness among older people and healthcare workers about frailty and its adverse outcome is critically important. Further longitudinal studies are needed to investigate underlying mechanisms between frailty and functional disability in older ages in Vietnam.

## Figures and Tables

**Figure 1:** Prevalence of individual frailty components.

**Figure 2:** Prevalence of participants having disability more than ≥3 IADL items and by component.

**Table 1:** Characteristics of the study sample by frailty status: robust, prefrail, and frail.

Characteristics	Overall	Frailty status			
		Robust	Prefrail	Frail	*p* value
*N* (%)	251 (100)	96 (38.2)	127 (50.6)	28 (11.2)	
Age (year, mean (SD))	84.6 (4.2)	83.6 (4.0)	84.8 (4.1)	87.2(4.5)	<0.01
Female	172 (68.5)	54 (56.2)	95 (74.8)	23 (82.1)	<0.01
Uncompleted high school	87 (34.7)	24 (25.0)	48 (37.8)	15 (53.6)	0.01
Married	140 (55.8)	61 (63.5)	65 (51.2)	14 (50.0)	0.15
Farmers	214 (85.3)	81 (84.4)	109 (85.8)	24 (85.7)	0.95
BMI levels					0.01
Underweight (<18.5 kg/m^2^)	74 (29.5)	18 (18.7)	50 (39.4)	6 (21.4)	
Normal weight (18.5-22.9 kg/m^2^)	132 (52.6)	59 (61.5)	57 (44.9)	16 (57.2)	
Overweight (≥23 kg/m^2^)	45 (17.9)	19 (19.8)	20 (15.7)	6 (21.4)	
Current smoking	18 (7.2)	12 (12.5)	5 (3.9)	1 (3.6)	0.04
Current drinking alcohol	53 (21.1)	27 (28.1)	22 (17.3)	4 (14.3)	0.09
Any chronic diseases	151 (60.2)	55 (57.3)	80 (63.0)	16 (57.1)	0.65
Living alone	12 (4.8)	1 (1.0)	10 (7.8)	1 (3.6)	0.06
≥3 IADL impairment	162 (64.5)	44 (41.1)	94 (67.1)	24 (85.7)	<0.01

BMI: body mass index; SD: standard deviation; IADL: Instrumental Activities of Daily Living.

The article "Association of Frailty Status and Functional Disability among Community-Dwelling People Aged 80 and Older in Vietnam" was published in 2021. Journal: Biomed Res Int.

**Table 2:** Association between frailty status and functional disability (≥3 IADL items) or each component IADL examined in separate models.

Frailty status	Adjusted^∗^ ORs (95% CI) of having disability								
	Combination	Single components							
	≥3 IADLs	Cooking	Housework	Laundry	Medication use	Manage money	Shopping	Tel use	Transport
Robust (ref)	1.0	1.0	1.0	1.0	1.0	1.0	1.0	1.0	1.0
Pre-frail	2.89 (1.58-5.29)	3.05 (1.65-5.65)	4.62 (1.93-14.51)	5.75 (2.33-14.20)	6.77 (3.16-14.20)	4.01 (1.65-9.71)	3.34 (1.79-6.21)	1.34 (0.70-2.57)	1.76 (0.95-3.25)
Frail	9.02 (2.37-34.33)	9.89 (2.37-11.25)	9.04 (2.44-33.56)	18.83 (4.29-82.58)	16.21 (4.42-59.46)	8.04 (2.14-30.13)	7.30 (2.11-25.31)	1.49 (0.39-5.69)	5.44 (1.70-17.42)

^∗^Adjusted for age, sex, education, marital status, occupation, BMI levels, current drinker, and having any chronic disease.

**Table 3:** Adjusted^∗^ ORs (95% CI) of having ≥3 IADL disability items by individual frailty components examined in separate models.

Frailty components	ORs (95% CI) of having ≥3 IADL disability items
Weight loss > 5%	1.14 (0.42-3.10)
Weak grip strength	1.43 (0.73-2.80)
Exhaustion	1.40 (0.65-3.02)
Low walking speed	4.21 (2.26-7.85)
Low physical activity	3.71 (1.68-8.19)

^∗^Adjusted for age, sex, education, marital status, occupation, BMI levels, current drinker, and having any chronic disease.

## Data Availability

The datasets of this study are available from the corresponding author on reasonable request.
